# Breast Lesions in Qassim Region, Saudi Arabia: A Retrospective Study

**DOI:** 10.7759/cureus.72050

**Published:** 2024-10-21

**Authors:** Reem Alsalamah, Emad Aljohani, Abdulaziz Altwijri, Faisal A Al-Harbi, Omar N Al-Harbi, Razan S Alharbi, Turki A Almutairi, Saleh M Alfadhel

**Affiliations:** 1 Surgery, Qassim University, Qassim, SAU; 2 College of Medicine, Prince Sattam Bin Abdulaziz University, Alkharj, SAU; 3 Breast and Endocrine Surgery, King Fahad Specialist Hospital, Buraydah, SAU; 4 College of Medicine, Qassim University, Buraydah, SAU

**Keywords:** benign, breast lesions, kfsh, ksa, malignant, qassim region

## Abstract

Introduction: A breast lesion is an unusual development in the breast tissue that typically appears as a lump or swelling. It encompasses a wide range of disorders, from benign to malignant, posing significant health challenges globally.

Methods: The study was a retrospective study conducted at King Fahad Specialist Hospital (KFSH), Buraidah, Qassim region in Saudi Arabia between March 10, 2017, and April 2, 2024. Data was cleaned, coded, and analyzed using SPSS version 27.

Results: The results revealed that most (639 (79.7%)) patients had symptomatic clinical presentations, with breast lump (470 (73.5%)) being the main presenting symptom. The majority (565 (70.4%)) of the patients presented malignant conditions, while 237 (29.6%) presented benign conditions. Of the patients who presented benign conditions, more than half (131 (55.3%)) were fibroadenoma benign lesions. Stage IIB cancer was the most common, constituting 192 (33.9%) of the patients. No complications were reported in the majority (480 (85.0%)).

Conclusion: The study revealed a considerably high prevalence of malignant conditions among patients. Fibroadenoma was the most common breast lesion type, followed by intra-ductal papilloma and benign phyllodes. Age and BMI were found to be the risk factors that predicted the development of breast cancers. Knowledge and awareness of the prevalence, risk factors, and treatment of breast illnesses, as well as early screening and diagnosis, promote better patient outcomes and healthcare delivery.

## Introduction

A breast lesion is an unusual occurrence in the breast tissue that ordinarily manifests itself as a lump or swelling [1]. Breast lesions can be benign (non-cancerous) or malignant (cancerous) and are typically found through physician assessment, mammograms, or self-detection [1]. While males are affected by breast lesions, the condition mainly affects females, with research indicating that at least 20% of females may develop breast lesions [2]. There are different types of lesions, including but not limited to cysts, adenosis, hyperplasia, lobular carcinoma in situ (LCIS), fibroadenomas, and radial scars. The different types of lesions have clinically different symptoms and carry other risks for developing cancer [3]. Although most of the breast lesions are benign, women with benign proliferative or atypical breast lesions are twice as likely to develop breast cancer in the Western world [4]. Furthermore, a study by Patil et al. (2024) determined that for every different type of benign breast lesion, there was a corresponding 25% increase in breast cancer risk after adjustment for age [5].

Given that the incidence rate of breast cancer in Saudi Arabia has grown almost 10-fold over the last two decades, it is essential to be thorough in evaluating and understanding the various risk factors, such as lesions [6]. According to the United States Preventive Services Task Force, mammography screening can be directly associated with a 22% reduction in cancer-related mortality for women aged 50 years and above and 15% in women aged between 40 and 49 [7]. Consequently, in the Western world, efforts aimed at fighting breast cancer have mainly focused on preventive interventions such as creating awareness and availing screening services, especially given that early identification and treatment lead to much better patient outcomes [8]. Similar cancer awareness campaigns in Saudi Arabia have been conducted to educate the public about various risk factors, such as self-examination of lesions, early detection, and mammography. Among patients with lesions, surgical evaluation through triple assessment, which involves clinical examination of the breast, mammography, and breast biopsy for histopathological confirmation, is necessary in many patients [9].

Despite the significant risk of breast cancer that breast lesions pose, there is insufficient research exploring the incident rate of breast lesions in Saudi Arabia. Region-based studies would create a basis for targeted and more accurate interventions and limit the possibility of developing breast cancer. Therefore, this retrospective study seeks to assess the prevalence of breast lesions among reproductive-age women in the Qassim Region, Saudi Arabia.

## Materials and methods

This study utilized a retrospective design, including all patients with breast lesions who underwent mastectomy at King Fahad Specialist Hospital (KFSH) in Buraidah, Saudi Arabia, between March 10, 2017, and April 2, 2024, and were residents of the Qassim region. The inclusion criteria for this study were patients who underwent mastectomy for breast lesions at KFSH in Buraidah, Kingdom of Saudi Arabia (KSA) and resided in the Qassim region. Conversely, the exclusion criteria encompassed patients with incomplete or missing medical records and those who underwent mastectomy as part of palliative care without curative intent.

This retrospective study utilized a non-probability convenience sampling technique whereby respondents were included in the completeness of their medical records. Cochrane sample size formula was employed to ascertain the sample size. The formula follows n = Z^2^p (1 − p)/d^2^. Where n represents the sample size, Z denotes the critical for 95% CI, 50% is the predetermined proportion, and d is the margin of error (5%). Initially, the minimum acceptable sample size computed was 384. However, to enhance the reliability of the study, we decided to include a larger sample size of 802 respondents.

The checklist (Table 6 of Appendices) specifically addressed the study's research questions and objectives. It included sections to capture essential information about patient demographics, clinical presentations, medical history, and management details. In the process of collecting secondary data, information was gathered from breast lesion patients who visited KFSH and were residing in the Qassim region. It involved accessing and reviewing existing medical records and data to ensure comprehensive and accurate information related to the patient's medical history and conditions.

Ethical approval was secured from the Qassim Ethics Committee (approval number 607/45/13634). One of the key ethical considerations was ensuring privacy by excluding personal identifiers, thereby preventing any association between individual identities and study results. Additionally, the respondents were fully informed about the study's purpose, procedures, potential risks, and benefits before voluntarily providing their consent, ensuring their participation was free from coercion.

Data analysis

After data collection, data cleaning commenced and involved identifying and removing outliers, duplicates, and incomplete entries. Once the data was cleaned, it was coded and imported into SPSS software version 27 (IBM Corp., Armonk, NY) for further analysis. Categorical variables were summarized using counts and frequencies. The associations between categorical variables were assessed using the Chi-square test, with a significance level set at p<0.05.

## Results

The study investigated 802 complete medical records of patients who underwent a mastectomy between March 10, 2017, and April 2, 2024, at KFSH in Buraidah, Saudi Arabia. The vast majority, 791 (98.6%) of the patients, were females, with only 11 (1.4%) of them being male. A considerable number, 211 (26.3%), of patients were aged 51-60 years. The great majority, 716 (89.3%) of the patients, were Saudi nationals; most, 667 (83.2%), of them were married, with a notable proportion (298 (37.2%)) of them being overweight (Table 1).

**Table 1:** Socio-demographic information of the patients (N=802)

Demographic information	Category	Frequency and proportion n (%)
Age	<30 years	96 (12.0%)
	30-40	141 (17.6%)
	41-50	208 (25.9%)
	51-60	211 (26.3%)
	>60 years	146 (18.2%)
Gender	Female	791 (98.6%)
	Male	11 (1.4%)
Nationality	Saudi	716 (89.3%)
	Non-Saudi	86 (10.7%)
Marital status	Single	108 (13.5%)
	Married	667 (83.2%)
	Divorced	16 (2.0%)
	Widowed	11 (1.3%)
BMI	Underweight	9 (1.1%)
	Normal	235 (29.3%)
	Overweight	298 (37.2%)
	Obese	172 (21.4%)
	Extremely obese	88 (11.0%)

Table 2 presents the patient's clinical history. Based on the record assessment, 289 (37.2%) patients had chronic disease. Of them, a considerable proportion (124 (42.8%)) had hypertension. Less than one-quarter, 135 (16.8%), of the patients had a family history of breast cancer, with 177 (22.1%) of them taking oral contraceptive pills. Most (639 (79.7%)) of the patients had symptomatic clinical presentations, with breast lump (470 (73.5%)) being the main presenting symptom for seeking medical attention. Nearly half of the patients presented symptoms on the left (321 (50.2%)), while 292 (45.7%) of them presented on the correct (292 (45.7%)) breast. A notable proportion (241 (37.7%)) of the patients took two to six months to have the presentation and reached medical attention, with the vast majority, 721 (89.9%), undergoing core needle biopsy. Most (565 (70.4%)) of the patients presented malignant conditions, while 237 (29.6%) presented benign conditions. Of the patients who presented benign conditions, 90 (38.0%) of them had a follow-up before; the great majority had received the surgical intervention (228 (96.2%)), as the result of the assessment with fibroadenoma (131 (55.3%)) being the final diagnosis.

**Table 2:** Patients’ clinical history

Clinical details	Categories	Frequency and proportion, n (%)
Chronic diseases?	Yes	289 (37.2%)
	No	504 (62.8%)
If yes, what is the chronic disease?	HTN	124 (42.8%)
	DM	91 (31.5%)
	Hyperthyroidism	4 (1.4%)
	Hypothyroidism	47 (16.3%)
	Iron-deficiency anemia	2 (0.7%)
	Renal failure	2 (0.7%)
	Asthma	17 (5.9%)
	Heart failure	2 (0.7%)
Family history of breast cancer?	Yes	135 (16.8%)
	No	667 (83.2%)
Patients taking OCPs?	Yes	177 (22.1%)
	No	625 (77.9%)
Clinical presentation?	Asymptomatic	2 (0.2%)
	Incidental	161 (20.1%)
	Symptomatic	639 (79.7%)
If symptomatic, what’s the main presenting symptom for seeking medical attention?	Breast lump	470 (73.5%)
	Axillary lump	11 (1.7%)
	Nipple discharge	36 (5.6%)
	Nipple deformity	12 (1.9%)
	Pain	97 (15.2%)
	Ulceration	10 (1.6%)
	Itching	3 (0.5%)
On which side is the presenting symptom?	Bilateral	26 (4.1%)
	Left	321 (50.2%)
	Right	292 (45.7%)
Time of having the presentation and reaching the medical attention?	<2 weeks	45 (7.0%)
	2 weeks-1 month	84 (13.2%)
	>1<2 months	40 (6.3%)
	2-6 months	241 (37.7%)
	>6 months<1 year	60 (9.4%)
	>=1 year	169 (26.4%)
Type of biopsy the patient underwent	Excisional	33 (4.1%)
	Core needle	721 (89.9%)
	FNA	8 (1.0%)
	Incisional	1 (0.1%)
	Lumpectomy	5 (0.6%)
	No biopsy	34 (4.3%)
Is the condition presented at the end benign or malignant?	Benign	237 (29.6%)
	Malignant	565 (70.4%)
There is a follow-up before?	Yes	90 (38.0%)
	No	147 (62.0%)
The end result of the assessment	Conservative and follow-up	9 (3.8%)
	Surgical intervention	228 (96.2%)
Final diagnosis?	Fibroadenoma	131 (55.3%)
	Fibrocystic	9 (3.8%)
	Benign phyllodes	28 (11.8%)
	Gynecomastia	1 (0.4%)
	Intra-ductal papilloma	39 (16.6%)
	Breast abscess	6 (2.5%)
	Mastitis	1 (0.4%)
	Ductal ectasis	1 (0.4%)
	Ductal hyperplasia	17 (7.2%)
	Epidermoid cyst	2 (0.8%)
	Lipoma	2 (0.8%)

Figure 1 below shows the frequency of various symptoms reported by patients. The most common symptom is a breast lump, experienced by nearly 73.5% of the patients. Pain is the second most common symptom, reported by around 15.2% of the patients. Other symptoms, such as nipple discharge, axillary lump, nipple deformity, ulceration, and itching, are significantly less common, each affecting less than 10% of the patients.

**Figure 1:** Bar graph depicting the frequency of breast cancer presenting symptoms

Table 3 illustrates the classification of breast cancer by the patients. Most of the patients, 565 (70.4%), presented malignancy. Of them, the histologic types included IDC (506 (89.6%)), with lesions presenting nearly equally on both the correct (279 (49.4%)) and left (277 (49.0%)) breasts. Most (192 (33.9%)) of the patients had stage IIB cancer. Molecular subtypes included positive ER (427 (75.5%)), positive PR (396 (70.1%)), and negative HER2 (385 (68.1%)). There were >20 (175 (31.0%)) Ki67 and inconclusive (247 (43.7%)) P53. Most of the patients took >6 months to five years (30 (76.1%)) to be diagnosed with breast CA. It was observed that 495 (87.6%) of the patients never completed the therapy. Only 70 (12.4%) completed the treatment. Of them, a notable proportion of (20 (28.6%)) of the patients had >3 years to five years after completing the therapy. Most (200 (35.4%)) of the patients underwent MRM surgery, with more than half, 319 (56.4%), having undergone sentinel lymph node biopsy-axilla surgery type. The majority, 480 (85.0%), of the patients had no surgery complications with only a few complications, which include seroma, 67 (11.9%); wound infection, 7 (1.2%); lymphedema, 6 (1.0%); and ecchymosis around the wound, 5 (0.9%).

**Table 3:** Characteristics of the breast cancer treatment outcomes among patients

Breast cancer characteristics	Categories	Frequency and proportion n (%)
Histologic types of breast cancer?	DCIS	23 (4.1%)
	IDC	506 (89.6%)
	ILC	18 (3.2%)
	IBC	4 (0.7%)
	Papillary carcinoma of the breast	3 (0.5%)
	Mucinous carcinoma of the breast	2 (0.3%)
	Malignant phyllodes tumor	1 (0.2%)
	No specific type	8 (1.4%)
Site of the lesion?	Right	279 (49.4%)
	Left	277 (49.0%)
	Bilateral	9 (1.6%)
Staging?	IA	34 (6.0%)
	IB	23 (4.1%)
	IIA	157 (27.8%)
	IIB	192 (33.9%)
	IIIA	67 (11.9%)
	IIIB	56 (9.9%)
	IIIC	19 (3.4%)
	IV	17 (3.0%)
Molecular subtypes (ER)	Equivocal	10 (1.8%)
	Negative	128 (22.7%)
	Positive	427 (75.5%)
Molecular subtypes (PR)	Equivocal	13 (2.3%)
	Negative	156 (27.6%)
	Positive	396 (70.1%)
Molecular subtypes (HER2)	Equivocal	58 (10.3%)
	Negative	385 (68.1%)
	Positive	122 (21.6%)
Ki67	<10	103 (18.2%)
	10-20	147 (26.0%)
	>20	175 (31.0%)
	Not available	140 (24.8%)
P53?	Positive	183 (32.4%)
	Negative	135 (23.9%)
	Inconclusive	247 (43.7%)
Time for diagnosing the patient with breast CA?	>1 month-6 months	5 (0.9%)
	>6 months-5 years	430 (76.1%)
	More than 5 years	130 (23.0%)
Patient completed the therapy?	Yes	70 (12.4%)
	No	495 (87.6%)
If yes, how long after completing the therapy?	≤1 year	25 (35.7%)
	>1 year-3 years	15 (21.4%)
	>3 years-5 years	20 (28.6%)
	>5 years	10 (14.3%)
The type of surgery underwent?	Lumbectomy	91 (16.1%)
	BCT	166 (29.4%)
	Simple mastectomy	101 (17.9%)
	MRM	200 (35.4%)
	Mastectomy with immediate reconstruction	4 (0.7%)
	Mastectomy with delayed reconstruction	3 (0.5%)
The type of axilla surgery underwent	Sentinel lymph node biopsy	319 (56.4%)
	Axillary dissection	193 (34.2%)
	SNL + axillary dissection	53 (9.4%)
Surgery complications?	None	480 (85.0%)
	Seroma	67 (11.9%)
	Wound infection	7 (1.2%)
	Lymphedema	6 (1.0%)
	Ecchymosis around the wound	5 (0.9%)

Table 4 depicts the patients’ breast cancer types by demographic characteristics. For benign, most of the cases were identified among patients aged <30 years (92 (95.8%)), singles (91 (84.3%)), underweight (6 (66.7%)), without chronic disease (179 (35.5%)), and those who had symptomatic clinical presentation (203 (31.8%)). For malignancy, most of the cases were also identified among patients aged >60 years (36 (93.2%)), divorced (14 (87.5%)), extremely obese (72 (81.8%)), those with chronic disease (240 (80.5%)), and those who had an asymptomatic clinical presentation (2 (100.0%)).

**Table 4:** Breast cancer types by demographic characteristics *Significant at p<0.05 level

Variable	Category	Benign	Malignancy	P-value
Age	<30 years	92 (95.8%)	4 (4.2%)	<0.001*
	30-40	61 (43.3%)	80 (56.7%)	
	41-50	49 (23.6%)	159 (76.4%)	
	51-60	25 (11.8%)	186 (88.2%)	
	>60 years	10 (6.8%)	136 (93.2%)	
Gender	Female	235 (29.7%)	556 (70.3%)	0.405
	Male	2 (18.2%)	9 (81.8%)	
Nationality	Saudi	223 (31.1%)	493 (68.9%)	0.04*
	Non-Saudi	14 (16.3%)	72 (83.7%)	
Marital status	Single	91 (84.3%)	17 (15.7%)	<0.001*
	Married	142 (21.3%)	525 (78.7%)	
	Divorced	2 (12.5%)	14 (87.5%)	
	Widowed	2 (18.2%)	9 (81.8%)	
BMI	Underweight	6 (66.7%)	3 (33.3%)	<0.001*
	Normal	94 (40.0%)	141 (60.0%)	
	Overweight	73 (24.5%)	225 (75.5%)	
	Obese	48 (27.9%)	124 (72.1%)	
	Extremely obese	16 (18.2%)	72 (81.8%)	
Chronic disease	Yes	58 (19.5%)	240 (80.5%)	<0.001*
	No	179 (35.5%)	325 (64.5%)	
Family history	Yes	35 (25.9%)	100 (74.1%)	0.186
	No	201 (30.1%)	466 (69.9%)	
Clinical presentation	Asymptomatic	0 (0.0%)	2 (100.0%)	0.020*
	Incidental	34 (21.1%)	127 (78.9%)	
	Symptomatic	203 (31.8%)	436 (68.2%)	

Table 5 presents the distribution of breast lesion types by demographic characteristics. For benign phyllodes, most of the cases were identified among patients aged 41-50 years (8 (16.7%)), married (19 (13.6%)), and overweight (12 (16.4%)). For fibroadenoma, most of the cases were identified among patients aged <30 years (73 (80.2%)), single (71 (78.0%)), and underweight (6 (100.0%)). For intra-ductal papilloma, most of the cases we found were among patients aged above 51 years old (10 (40.0%)), divorced (2 (100.0%)), and extremely obese (6 (37.5%)). Other cases comprised patients mostly aged 51-60 years (7 (28.0%)), married (31 (22.1%)), and extremely obese (4 (25.0%)). For Saudi residents, the prevalence rate of fibroadenoma was 130 (55.8%) followed by intra-ductal papilloma (36 (16.2%)) and benign phyllodes (27 (12.2%)).

**Table 5:** Distribution of breast lesion types by demographic characteristics *Significant at p<0.05 level

Variable	Category	Benign phyllodes	Fibroadenoma	Intra-ductal papilloma	Others	P-value
Age	<30 years	10 (11.0%)	73 (80.2%)	3 (3.3%)	5 (5.5%)	<0.001*
	30-40	6 (9.8%)	34 (55.7%)	4 (6.6%)	17 (27.9%)	
	41-50	8 (16.7%)	15 (31.3%)	17 (35.4%)	8 (16.7%)	
	51-60	3 (12.0%)	5 (20.0%)	10 (40.0%)	7 (28.0%)	
	>60 years	1 (10.0%)	3 (30.0%)	4 (40.0%)	2 (20%)	
Gender	Female	28 (12.0%)	130 (55.8%)	37 (15.9%)	38 (16.3%)	0.571
	Male	0 (0.0%)	1 (50.0%)	1 (50.0%)	0 (0.0%)	
Nationality	Saudi	27 (12.2%)	125 (56.3%)	36 (16.2%)	34 (15.3%)	0.522
	Non-Saudi	1 (7.7%)	6 (46.2%)	2 (15.4%)	4 (30.8%)	
Marital status	Single	9 (13.6%)	71 (78.0%)	4 (4.4%)	7 (7.7%)	<0.001*
	Married	19 (13.6%)	59 (42.1%)	31 (22.1%)	31 (22.1%)	
	Divorced	0 (0.0%)	0 (0.0%)	2 (100.0%)	0 (0.0%)	
	Widowed	0 (0.0%)	1 (50.0%)	1 (50.0%)	0 (0.0%)	
BMI	Underweight	0 (0.0%)	6 (100.0%)	0 (0.0%)	0 (0.0%)	<0.001*
	Normal	10 (10.6%)	65 (69.1%)	8 (8.5%)	11 (11.7%)	
	Overweight	12 (16.4%)	40 (54.8%)	8 (11.0%)	13 (17.8%)	
	Obese	5 (10.9%)	15 (32.6%)	16 (34.8%)	10 (21.7%)	
	Extremely obese	1 (6.3%)	5 (31.3%)	6 (37.5%)	4 (25.0%)	

## Discussion

A female preponderance constituting 791 (98.6%) of all the patients with breast cancer in the Qassim region, Saudi Arabia, revealed a high prevalence of breast cancer among old age patients, with more than 65% of the patients belonging to the over 41 years age groups. A similar study conducted in the Qassim region by Akhtar et al. noted a higher prevalence of breast cancer in patients aged 40 years and above [10]. The survey conducted by Al-Rikabi et al. reported an 18% prevalence of breast cancer among patients aged less than 40 years, which is lower than our study, which revealed a 237 (29.6%) prevalence of breast cancer among patients aged less than 40 years [11]. This variation may be due to differences in varied dietary and cultural practices, lifestyle changes, and exposure to some environmental carcinogens [12].

It was observed that a considerable number, 289 (37.2%), of patients had a chronic disease, with nearly half, 124 (42.8%), with HTN. In a study conducted by Kang et al., chronic diseases were reported in less than half of the cancer patients in the study, with hypertension, hyperlipidemia, and diabetes being the most common [13]. In the current study, patients who had a family history of breast cancer constituted less than one-quarter of 135 (16.8%) of the patients. The common clinical presentation was symptomatic (639 (79.7%)), with breast lump (470 (73.5%)) being the main presenting symptom for seeking medical attention. Breast lump was also reported as the most prevalent symptomatic clinical presentation in the study conducted by Saggu et al. in Saudi Arabia [14]. Nearly half of the patients presented symptoms on the left breast, 321 (50.2%), while 292 (45.7%) of them presented on the right breast, with the majority, 721 (89.9%), of them undergoing core needle biopsy. 

Malignant condition was the most prevalent type, constituting 565 (70.4%) of the patients, while benign conditions were represented by 237 (29.6%) of the patients. Of the patients who presented benign conditions, 90 (38.0%) of them had a follow-up before, with a predominance of fibroadenoma benign lesions (131 (55.3%)), which is in line with Zhu et al.’s findings that reported high incidences of fibroadenoma benign tumors among women aged 18-40 years in Guangdong province in China [15]. 

The most frequent histologic type was invasive ductal carcinoma (506 (89.6%)), which manifested in the form of lesions and presented on both breasts in patients with malignancy conditions. Furthermore, stage IIB cancer was the most common, constituting 192 (33.9%) of the patients, with frequent molecular subtypes being positive ER (427 (75.5%)), followed by positive PR (396 (70.1%)), and then negative HER2 (385 (68.1%)). 

The benign condition was found to be common among patients aged <30 years (92 (95.8%)) and underweight (6 (66.7%)) while the malignant condition was prevalent among patients aged >60 years, extremely obese (72 (81.8%)) and having a chronic disease (240 (80.5%)). These findings are reinforced by Dubey et al., who reported a significant association between breast lesion malignancy and advancement of age and the existence of underlying conditions among the patients [16]. Similarly, higher cases of benign conditions were reported among patients aged 35 years and below in a study conducted by Alghamdi et al., consistent with the current study [17]. The most prevalent breast lesion type was a fibroadenoma, with most of its cases identified among patients aged <30 years (73 (80.2%)), single (71 (78.0%)), and underweight (6 (100.0%)), followed in descending order by intra-ductal papilloma, with most of the cases identified among patients aged above 51 years old (10 (40.0%)), divorced (2 (100.0%)), and extremely obese (6 (37.5%)) and finally, benign phyllodes, with most of the cases identified among patients aged 41-50 years (8 (16.7%)), married (19 (13.6%)), and overweight (12 (16.4%)). The findings are reinforced by Najjar et al., who reported fibroadenoma to be the most frequent breast lesion type among cancer patients, with age and BMI as the risk factors that predict the development of cancer, which is in agreement with our current findings [18]. 

The major limitation of this investigation is the fact that the nature of the collected data and information regarding the breast lesions were extracted from the patient's records and files; the absence of detailed data on the grading and staging of breast cancers as well as the subsequent management poses significant constraints on the achievement of the study objectives. 

## Conclusions

The study revealed a considerably high prevalence of malignant conditions among patients who attended KFSH in Buraidah, Qassim region in Saudi Arabia, between March 2017 and April 2024. Fibroadenoma was found to be the most common breast lesion type, followed by intra-ductal papilloma and benign phyllodes. Age and BMI were found to be the risk factors that predicted the development of breast cancers. Knowledge and awareness of the prevalence, risk factors, and treatment of breast illnesses, as well as early screening and diagnosis, promote better patient outcomes and healthcare delivery.

## Appendices

**Table 6:** Checklist

Question	Options
Age?	<30 years, 30-40 years, 41-50 years, 51-60 years, >60 years
Gender?	Male, female
Nationality?	Saudi, non-Saudi
Marital status?	Single, married, divorced, widowed
BMI?	Underweight, Normal, Overweight, Obese, Extremely Obese
Chronic diseases?	Yes, no
If yes, what is the chronic disease?	HTN, DM, hyperthyroidism, hypothyroidism, iron-deficiency anemia, renal failure, asthma, heart failure
Family history of breast cancer?	Yes, no
Patient taking OCPs?	Yes, no
Clinical presentation?	Symptomatic, incidental
Main presenting symptom for seeking medical attention?	Breast lump, axillary lump, nipple discharge, nipple deformity, pain, ulceration, itching, features of metastasis
On which side is the presenting symptom?	Right, left, bilateral
Time from presentation to medical attention?	<2 weeks, 2 weeks-1 month, >1<2 months, 2-6 months, >6 months<1 year, ≥1 year
Type of biopsy performed?	Excisional, core needle, FNA, incisional, lumpectomy, no biopsy
Is the condition benign or malignant?	Benign, malignant
Is there a follow-up?	Yes, no
End result of assessment?	Conservative and follow-up, surgical intervention
Final diagnosis for benign lesions?	Fibroadenoma, fibrocystic, benign phyllodes, gynecomastia, intra-ductal papilloma, breast abscess, mastitis, ductal ectasia, ductal hyperplasia, epidermoid cyst, lipoma
Final diagnosis for malignant lesions?	DCIS, LCIS, IDC, ILC, IBC, papillary carcinoma, mucinous carcinoma, malignant phyllodes, angiosarcoma, lymphoma
Site of lesion?	Right, left, bilateral
Staging of breast cancer?	IA, IB, IIA, IIB, IIIA, IIIB, IIIC, IV
Molecular subtypes of cancer?	ER (positive, negative, equivocal), PR (positive, negative, equivocal), HER2 (positive, negative, equivocal)
Ki67 test result?	<10, 10-20, >20, not available
P53 test result?	Positive, negative, inconclusive
Time of diagnosis of breast cancer?	≤1 month from now, >1 month-6 months, >6 months-5 years, >5 years
Has the patient completed the therapy?	Yes, no
If yes, how long after completing therapy?	≤1 year, >1 year-3 years, >3 years-5 years, >5 years
Type of surgery performed?	Lumpectomy, BCT, simple mastectomy, MRM, mastectomy with immediate reconstruction, mastectomy with delayed reconstruction
Type of axilla surgery performed?	Sentinel lymph node biopsy, axillary dissection, SLN + axillary dissection
Surgery complications?	None, seroma, wound infection, lymphedema, ecchymosis around the wound
